# Individual Online Learning Behavior Analysis Based on Hadoop

**DOI:** 10.1155/2022/1265340

**Published:** 2022-09-08

**Authors:** Ning Xiang

**Affiliations:** School of Journalism and Communication, Hunan Mass Media Vocational and Technical College, Changsha 410100, China

## Abstract

The online individual behavior analysis is an important means for mining user interests. The user retweeting behavior prediction is typical problem for online individual behavior analysis. In order to make online learning behavior prediction method more suitable for the application of large-scale datasets, the improved condensed K nearest neighbor (ICKNN) method is proposed in this paper. Inspired by the idea of compressing samples in the condensed nearest neighbor (CNN) algorithm, this proposed method has adopted the Hadoop platform to parallelize the traditional CNN algorithm. For the traditional CNN method, as the value of K increases, the compression ratio decreases and so as the efficiency. The proposed ICKNN method can parallelize the traditional CNN method under the Hadoop framework to enhance efficiency. The proposed ICKNN method in this paper is validated by actual Twitter retweeting dataset. It can be seen that the proposed method in this paper has a higher compression rate than the traditional CNN algorithm. In terms of accuracy, the classification accuracy of the proposed ICKNN method has decreased compared with the traditional KNN method. However, the time consumed by the ICKNN method has significantly reduced compared with the traditional KNN method and CNN method, which can greatly improve the efficiency.

## 1. Introduction

As the access of Internet technology is not limited by time and space, and as it has the feature of low cost and fast information transmission, it has quickly become one part of people's daily lives. Due to the rapid development of the Internet, social network has become ubiquitous. The massive data volume on social media can provide fundamental support for data-related researches, and valuable information can be achieved from data mining, which can be useful for individuals, enterprises, and governments [1, 2]. Under the condition of massive data volume, traditional methods relying only on a single computer have the disadvantages of low efficiency and significant processing latency. Therefore, traditional data mining methods need to be improved to meet the requirements under the condition of big data.

Under current conditions, an important profit model for social networks is to predict the user interests for content promotion according to users' behavior. In order to mine users' interests, it is feasible for online predicting the online learning behavior of individual users. Online learning behavior prediction can enable the study of the transmission mechanism, diffusion mode, and related characteristics of users' tweets, which can provide users with personalized services and enable strategic marketing. Moreover, necessary information from the public social network platform can be obtained for making strategies for the related companies [3, 4]. As a matter of fact, individual online learning behavior analysis and prediction is now a hot research topic.

For the prediction of online learning behavior, the authors in literature [5] have firstly applied the classification algorithm to the area. The content of the microblog is represented by a feature vector and with the number of 0 and 1 to indicate whether a tweet is forwarded. Herein, the retweeting prediction problem can be transformed to a corresponding pattern recognition problem. Current methods for online learning behavior prediction are mainly two folds: (1) the first aspect is to enable more effective establishment of features in the content of the microblog for classification, i.e., the feature-centric methods [6–9]. (2) The second aspect is to build a better classification model to predict whether a tweet is forward or not, i.e., the classifier-centric methods [10–13]. The following will give introductions of the online learning behavior prediction methods according to the two types of methods mentioned above. In feature-centric methods, it is verified in literature [14] that different features may have a significant impact on the performance. In literature [15], the correlation features between users and their posts are extracted and adopted. It is proved that the correlation features can greatly improve the performance of prediction compared adopting either just user features or just features from the content of the tweets. The authors have added new features to the feature vector, for example, the interaction frequency between the current user and the upstream user, and the feature vector of the upstream user. Thus, the accuracy of online learning behavior can be improved. Similarly, the authors in literature [16] have taken consideration of hot topics and transmission characteristics when establishing the feature vector, which have also improved the accuracy of prediction.

For the classifier-centric methods, in [17], the random walk modeling is applied for the calculation of forwarding probability from the multi-dimensional feature vectors, so as to predict the online learning behavior. In literature [18], the support vector machine (SVM) classifier is adopted. In this literature, SVM is firstly adopted to train an unweighted model, from which the importance of different dimensions of the features is obtained. The importance can be adopted as the feature weights. In this paper, it is proved that blog posts with positive emotions have a greater probability of forwarding than blog posts with negative emotions. The authors in [19] have also adopted SVM for classification, where feature combination method has been applied to verify the importance of different features for online learning behavior prediction. In [20], the forwarding behavior is predicted by adopting a random forest classifier. Specifically, it has adopted the information gain method to make use of three types of features, including user-based, relationship-based, and topic-based features. As a result, the problem of imbalance samples is solved by using the oversampling technology for retweeting prediction. In literature [21], the feature-centric and classifier-centric methods are combined, and the online learning behavior is predicted through multi-task learning. The authors in [22] go a step further and take the relationship between different tasks into consideration to improve the prediction accuracy.

Under the background of massive data, traditional data mining methods need to be migrated to such an environment. Hadoop is a big data ecosystem, which can provide an overall solution to large-scale data analysis [23–25]. The core components of Hadoop are the Hadoop Distributed File System (HDFS) and the MapReduce paralleled programming model. The existence of HDFS makes Hadoop capable of storage for large amounts of data in a distributed way. And the existence of MapReduce ensures that Hadoop is efficient for parallel computing. The HDFS is one of the core components of the Hadoop architecture. It can be adopted to store large files. Sometimes, if the size of the file exceeds the capacity of a single computer, HDFS can be used to store the data in a distributed manner on several computers or servers, and the files can then be processed by locating and finding through the directory tree [26–28]. The MapReduce distributed computing framework is suitable for parallel computing in a distributed environment with high availability deployment at multiple servers. It is also one of the core components of the Hadoop system. The core idea is to make use of the distributed large-scale file data in the HDFS system. By dividing the task into multiple MapReduce sub-tasks for parallel processing, data operations for a large-scale data volume can be reached, even at the TB or PB level [29–31]. Over all, the Hadoop framework has the following advantages: (1) it has better capacity expansion feature; (2) the cost is low, and the framework can meet the computing requirements with only several ordinary computers; (3) the application of HDFS enables the system to have high data reliability; (4) the application of MapReduce makes large-scale data processing more efficient.

In order to make online learning behavior prediction method more suitable for the application of large-scale datasets, the improved condensed K nearest neighbor (ICKNN) method is proposed in this paper, which can be adopted to solve the problem of reduced classification efficiency in the context of big data. In the proposed method, a consistent sample subset from the original sample set is firstly obtained according to a reasonable decision boundary, so as to achieving the goal of compressing sample numbers and improving classification efficiency. Generally speaking, in order to improve the compression ratio of the algorithm, that is, to improve the efficiency of the algorithm, it is necessary to reduce the *k* value in the algorithm, which is the number of neighbors. However, when *k* = 1, which is the smallest value, the robustness of the classification can be degraded greatly. Therefore, the value of *k* takes a larger value herein at the cost of a smaller compression ratio. In this paper, in order to further improve the compression ratio of the algorithm and to improve the efficiency, the traditional condensed nearest neighbor (CNN) algorithm is parallelized in the framework of Hadoop. After parallelizing the original CNN algorithm, the proposed method is verified by the actual microblog dataset. The experimental results show that the ICKNN algorithm in this paper implemented on the Hadoop platform has a better compression rate than the traditional CNN algorithm, while the prediction performance is better with a higher classification accuracy.

## 2. Methods

In the proposed method, after parallelizing the traditional CNN method [32], it can be implemented at the Hadoop big data framework. The results show better retweeting prediction performance with a better algorithm compression ratio, which can effectively improve the computational efficiency. In this section, the basics of the Hadoop framework is introduced at first, then the CNN method is introduced, and at last the descriptions of how to parallelize the CNN method and implement it to the Hadoop framework are introduced.

### 2.1. Introduction of the Hadoop Framework

Hadoop is an overall solution for processing large-scale data analysis. Traditional databases are only suitable for processing structured data, such as query using Structured Query Language (SQL) statements, while Hadoop can process structured, semi-structured, and unstructured data from different sources and formats. It has backup in storage and can be dynamically expanded. For processing queries, the Hive statements can be adopted.

The core components of the Hadoop framework are the HDFS and the MapReduce parallel programming model. The existence of HDFS makes Hadoop capable of distributed storage of large amounts of data. The existence of MapReduce ensures that Hadoop is good at efficient parallel computing. The two core components of the Hadoop framework, HDFS and MapReduce, are introduced as follows.

The HDFS supports one-time writing and unlimited reads, and the already written cannot be modified. HDFS is one of the core components of the Hadoop architecture. It can be adopted to store large files. When the size of the stored files exceeds the capacity of a single machine, HDFS can be adopted to store the data in a distributed manner on several computers, and the stored files can be located by the directory tree. The illustrational principle of the mentioned HDFS principle is shown in Figure 1.

HDFS has the following advantages: (1) HDFS supports the storage of large files, with even TB or PB size, and can process tens of thousands of nodes at the same time. (2) The HDFS system is suitable for big data processing. The NameNode is responsible for the management of the file directory tree and the mapping information of data blocks. This can make fast location of the data block [27]. (3) The backup strategy adopted by HDFS is usually twice backup, which are stored in different DataNodes. If a data block is broken, the internal mechanism of HDFS will automatically adopt the backup data to repair it. With this type of data repairing capacity, the HDFS framework can be deployed on relatively cheaper servers. Once the data are lost or interrupted, it can be quickly retrieved.

The MapReduce is also one of the core components of the Hadoop system. It is a distributed computing framework which is suitable for deployment at a distributed environment composed with several servers with high availability. The core idea is to make use of the distributed large-scale file data in the HDFS system. By dividing the task into multiple MapReduce sub-tasks for parallel processing, data operations for a large-scale data volume can be reached, even at the TB or PB level [30]. Similar to the HDFS system, MapReduce has also adopted a master-slave architecture, where the NameNode is responsible for the coordination and control of tasks, including task initialization, assignment, and communication with DataNodes. The DataNode then is responsible for performing the Map and Reduce slicing tasks, and asking the NameNode for the required file information during the processing. The MapReduce can be divided into four stages, including data slicing, mapping stage, shuffle stage, and the combine stage. The processing flowchart of the MapReduce framework is shown in Figure 2.

The MapReduce task is processed with the following stages: (1) at the start of the task, the client sends a Job ID assignment request to the task assignment NameNode. (2) The NameNode returns the Job ID to the client, and the client copies the JAR file package, configuration policy file, and file slice information required for task execution to the job queue of the NameNode node of HDFS. (3) The NameNode schedules the tasks in the job queue, creates a map task for a single job, and assigns it to the DataNode execution node which contains the data blocks processed by the map. (4) After all tasks are executed, NameNode sets the task to “completed state,” and the client queries that the NameNode state is “completed,” and sends a message to inform the user.

MapReduce has the following advantages: (1) nodes are easy to expand. When cluster resources are insufficient, the nodes can be expanded for computing. (2) The resources are easy to coordinate and have strong fault tolerance. When a node failure causes the calculation to fail, other nonfaulty nodes can be adopted for calculation. (3) Parallel computing is adopted, which is suitable for TB or even PB-level data processing.

### 2.2. The CNN Algorithm

In the traditional K nearest neighbor (KNN) algorithm, each time to determine a sample's type, all samples are traversed. Therefore, the classification efficiency will decrease significantly with an increase of training samples. To solve the problem of reduced efficiency, the condensed nearest neighbor (CNN) algorithm is proposed in [32], which can effectively reduce the number of samples required for classification. In the CNN algorithm, it is believed that the closer a sample is to the decision boundary, the greater the impact it has on the classification results and vice versa. Therefore, the classification problem can be attributed to the problem of obtaining the sample points with the smallest distance from the decision boundary, and at the same time removing the sample points that are far away.

Before the description of the CNN algorithm, a classification model should be established at first. Assuming that *S* denotes the training set, the number of samples is *N*, and it should be divided into *C* classes, the sample set can be expressed as

(1) $$\begin{array}{c} S=\left\{S_{1}^{N_{1}},S_{2}^{N_{2}},...,S_{C}^{N_{C}}\right\}\text{.} \end{array}$$

Among them, *S*_*i*_^*N*_*i*_^ represents the sample set from *i* th class in *S*, and the number of sample points contained is *N*_*i*_; then, the sample can be expressed as

(2) $$\begin{array}{c} S_{i}^{N_{i}}=\left\{s_{i}^{p}\right\},i=1,2,...,C\;,p=1,2,...,N_{i}\text{,} \end{array}$$

where

(3) $$\begin{array}{c} \overset{C}{\underset{i=1}{\sum }}N_{C}=N\text{.} \end{array}$$

Then, the set of *k* nearest neighbors found can be expressed as

(4) $$\begin{array}{c} T_{knn}{\left(s_{i}^{q}\right)}_{j}=\left\{x_{1},x_{2},...,x_{k}\right\}\text{,} \end{array}$$

*T*_*knn*_(*s*_*i*_^*q*^)_*j*_ denotes the sample set of class in *i* with samples found in class *j* with *k* nearest neighbor.

For each sample, a corresponding decision influence factor *U*_affect_ is assigned, which is determined by the location of the samples. If the decision influence factor is large, it means that the distance between the sample point and the classification decision boundary is closer. The set of decision influence factor can be expressed as

(5) $$\begin{array}{c} U_{affect}=\left\{u_{affect,1},u_{affect,2},...,u_{affect,c}\right\}, \end{array}$$

where *u*_affect,*n*_ represents the decision influencing factors of all samples in category *m*, and *u*_affec*t*,1_[*i*] represents the decision influencing factors of sample *i* within.

The flow of the CNN algorithm is shown as follows.

1. Iterate over the number of categories *C*.
2. In each type *c*, iterate over the samples in the sample set of *S*_*c*_^*N*_*c*_^.
3. Get the *k* nearest neighbors for the sample *s*_*i*_ among other types and get *T*_*knn*_(*s*_*i*_)={*x*_1_, *x*_2_, *x*_*k*_}.
4. The corresponding decision influence factors are added by 1.
5. Delete the samples whose decision influence factors are less than 1 and get the consistent subset *S*_min_^*i*^.
6. Perform the normal KNN algorithm over *S*_min_^*i*^ and the classification result.

In the CNN algorithm, the value of *k* is an important factor affecting the compression rate of the CNN algorithm. If *k* equals to 1, the compression rate of the algorithm is relatively high. After the compression, only the samples which are near to the boundary are remained. In this condition, the classification performance can be degraded if the number of samples has been decreased too much. If the value of *k* is relatively large, samples which are farther away from the boundary can be remained. In this case, the compression rate will decrease. If all samples are remained in the set, then the compression rate is 0.

### 2.3. The ICKNN Algorithm Implemented on Hadoop

According to the mentioned CNN algorithm, when *k* is not equal to 1, its algorithm compression ratio is still unsatisfactory, and when the training dataset is large, there is still a problem of low computational efficiency. In order to improve computing efficiency, a parallel computing method is designed for the CNN algorithm, here noted as IKCNN, and is implemented adopting the MapReduce framework.

It is found that the calculation of *k* nearest neighbors of each category is independent. As a result, the parallelized calculation can be implemented. If the sample points in the sample set can be divided into *C* categories, then the number of computing threads can also be set to *C*. With *C* threads computing at the same time, the speed can be accelerated significantly.

The MapReduce framework is implemented in this paper for the ICKNN algorithm. The format of data storage is <key, value>, which is key-value paired. As mentioned, it is necessary to allocate the calculation tasks to each sub-nodes and integrate the calculation results from each node to obtain the final result. In the process, Map and Reduce are processed in parallel, which can be independent and efficient. The final output is acquired by the Reduce function. According to the processing flow of by MapReduce, three jobs are formed which can be serially executed. In our paper, the three jobs are named as job A, job B, and job C. Among the jobs, job A is related to the calculation process of nearest neighbors. Job B obtains the *k* nearest neighbors with their corresponding influence factors based on the results of job A. If the influence factor is bigger than zero, it is taken out and saved. Job C aggregates the previous results to form the final compressed training set. The three jobs are described as follows, respectively.

In job A, the Mapper class, Combiner class, and Reducer class are included. The functions of each class are different. The Mapper class divides the training sample set into multiple splits and assigns them to different map tasks.

The Mapper class is mainly adopted to calculate the distance between samples in the training set. Then, the Combiner class is adopted to aggregate the obtained results. Both of these two classes are run in a DataNode, which can process the data directly without the need of transmitting data, thus is more efficient. In addition, the Combiner class can also reduce the cost of data transmission from the Mapper class, which will save much time in data transmission. The Reducer class can further process the output of the Combiner class, and after summarizing these results, *k* global nearest neighbor samples of non-self-category class in the training set can be obtained. The process of job A is shown in Figure 3.

For the Combiner class, the input of the Combiner class is the value list corresponding to the output key of the Mapper class. The Reduce function compares the distances of sample points in the value list and then saves the *k* values with the smallest distances in the local *k* nearest neighbor set. It is worth noting that the Combiner class is essentially a Reducer class, and it runs locally. Each Combiner class has a corresponding Mapper class, so the local *k* nearest neighbor sample point set output by the Combiner class is only the local *k* nearest neighbors in the block.

For the Reducer class, the execution process of the Reducer class is basically the same as the Combiner class. The value corresponding to the output key of the Combiner class needs to be merged, so as to obtain the input to the Reducer class.

For the work of job B, a new hash table in the Mapper class is built at first, where its key and value should be set. In our implementation, the key is the ID of the samples, and the value is the number of *k* nearest neighbors (with other categories) of the corresponding sample ID, which is obtained from the results of job A. Here, the output format of job A is shown as follows: Category-id1 to id *k*. To read the file in this format, the TextInputFormat format is adopted. The input format of the map is <line number, line text>, where the line text has the mentioned format of Category-id1 to id *k*. The line text can be processed to *k* + 1 substrings and is stored in linestr. Then for each id in linestr, the corresponding keys are obtained, which is the ID number plus 1. With the key, it is added to the hash table again. If the key corresponding to the ID cannot be obtained, then the key-value of (id, 1.0) is directly added to the hash table. The above steps have handled the input data. After the processing completed, the *k* nearest neighbors of all samples belonging to other categories have been stored in the hash table. After the above process, the calculation of the influence factor of each sample is completed. Then after sorting, the IDs of the samples whose influence factors are greater than or equal to 1 can be obtained. The processing flow is shown in Figure 4.

For processing flow of job C, only the Mapper class is included. The initialization is performed by adopting the results of job B as the configuration information. Then, the setup() function of the Mapper class is overloaded and the ID array based on the output of job2 is initialized. Then, the output file from job B is read, and the index array is initialized, which is adopted to store the reserved sample IDs. If the index array includes the input sample ID, it outputs directly.

## 3. Experimental Results

In this paper, the tweet dataset from [33] is used to evaluate the basic performance of the proposed method. Accordingly, the performance of the proposed method for online learning behavior prediction can be evaluated. In this dataset, there are 436,330 posts that can be forwarded and the attributes of the dataset are shown in Table 1. This part in the dataset can be directly adopted for predict the online learning behavior. Noting that in the dataset, there are some posts which cannot be adopted, including the commenting posts. The construction of a sample is to find out the user's following users based on the user-following relation network constructed by the user_friends table. Then based on the tweet_info table, whether the following users have retweeted the post can be found. The construction of the retweeting information is as follows: (1) build the index list of [userId, (friendsId1,…, friendsId*n*)] on the user_friend table and the list of [userId, (tweetId1,…, tweetId*k*)] on the tweet_info table. (2) If a retweeted post is obtained, find user A and the creation time *T* of the pos. (3) According to user A in [userId, (friendsId1,…, friendsId*n*)], find out the corresponding follower user B. (4) According to [userId, (tweetId1,…, tweetId*k*)], find out all the blog post IDs of B. (5) Select the non-retweeted post corresponding according to the creation time *T*, and combine user A's own original post at time *T*; the retweeting data samples can be obtained. In addition to the above basic attributes, the number of retweets obtained from tweet_info, the user obtained from user_info, and the user attributes can also be obtained.

After obtaining the relevant data, other procedures are implemented to make the samples more applicable for processing. The data are preprocessed by missing value handling, user cleaning, etc. Then, the relevant features for classification are built. The constructed features can be divided into three categories: user-related feature group, post-related feature group, and context-based feature group. The user-related feature groups are from the perspective of users, including a series of characteristics of the users themselves. The blog-related feature groups are from the perspective of the contents of the tweets. The context-based feature group is a series of feature descriptions of the situations faced by the user.

### 3.1. Related Metrics of the Method

To better evaluate the proposed method in this paper, proper metrics are needed. The confusion matrix for a common binary classification problem is shown in Table 2.

From the table, the accuracy metric can be derived. The accuracy metric represents the probability that the samples can be accurately classified. It is actually the ratio of the correctly classified samples to the total samples.

(6) $$\begin{array}{c} Acc=\frac{TP-TN}{N}\text{.} \end{array}$$

In addition to the metric related to classification, there is also a special indicator in this paper, that is, the algorithm compression ratio. For KNN typed algorithms, the algorithm compression ratio can be expressed as

(7) $$\begin{array}{c} CR=\frac{N-N_{c}}{N}\text{,} \end{array}$$

where *N* represents the number of samples in the original sample set and *N*_*c*_ represents the number of samples after compression. According to the evaluation metrics in this section, the proposed prediction method in this paper can be evaluated.

### 3.2. Comparisons of Different Methods

In order to verify the proposed method in this paper, experiments are carried out adopting the mentioned retweeting dataset. The proposed ICKNN method is compared with the common KNN method and the CNN method. Figure 4 and Table 3 respectively, show the compression ratio, accuracy of the KNN algorithm, and CNN algorithm when the *k* values are different. According to the results in Figure 5 and Table 3, it can be seen that as K increases, in general, the compression ratio decreases. The blue bar denotes the accuracy, and the yellow bar denotes the compression rate. It can also be seen that the proposed method in this paper has a higher compression ratio than that of the traditional CNN algorithm under the both conditions when *k* = 1 and *k* = 2. In addition, in terms of accuracy, under the conditions of *k* = 1 and *k* = 2, the ICKNN method proposed in this paper has a lower classification accuracy than the traditional KNN method, because in the classification process, only the nearby samples around the classification boundary are remained. However, compared with the traditional CNN algorithm, the accuracy of the ICKNN algorithm has still improved with a higher compression ratio. It can be seen from Table 3 that compared with the traditional CNN algorithm, the proposed method has improved the compression ratio by 3% and the accuracy by 52% under the condition of *k* = 1. Under the condition of *k* = 2, the compression ratio has improved by 8%, and the accuracy has improved by 14%.

Since the proposed ICKNN method in this paper can be run in parallel under the Hadoop platform, in addition to the sample compression ratio, it can still reduce the running time and improve the classification efficiency. The different time costs of the different methods are shown in Table 4. The time cost of classification by the proposed ICKNN method, CNN method, and KNN method is 420s, 429s and 308s, respectively. Here, the proposed ICKNN method in this paper is run under the Hadoop platform with 4 nodes. It can be seen that compared with the traditional KNN method and CNN method, the time consumed by the ICKNN method has reduced by 36% and 28%, respectively, which can greatly improve the classification efficiency.

## 4. Conclusions

The online learning behavior prediction is a typical problem for online learning of individual behavior. In order to make online learning behavior prediction method more suitable for the application of large-scale datasets, the ICKNN method is proposed in this paper. The proposed method has adopted the Hadoop platform to parallelize the traditional CNN algorithm to boost classification efficiency. The proposed ICKNN method in this paper is validated by the actual Twitter retweeting dataset. It can be seen that the proposed method in this paper has increased the compression rate by 3% and 8% than the traditional CNN algorithm under the conditions of *k* = 1 and *k* = 2, respectively. In addition, in terms of accuracy, under the conditions of *k* = 1 and *k* = 2, the classification accuracy of the proposed ICKNN method has decreased compared with the traditional KNN method. Compared with the traditional KNN method and CNN method, the time consumed by the ICKNN method has reduced by 36% and 28%, respectively, which can greatly improve the classification efficiency. The current results are acquired under the condition that the number of nodes of the Hadoop framework is four. For other number of nodes, it will be studied in our future work.

## Figures and Tables

**Figure 1:** An illustrational principle of how the HDFS works.

**Figure 2:** The processing flow of the MapReduce framework.

**Figure 3:** The flowchart of the mapper implementation in job A.

**Figure 4:** The flowchart of mapper class implementation in job B.

**Figure 5:** The different accuracy and compression rate of the proposed ICKNN, the KNN, and the CNN method.

**Table 1:** Some attributes of the retweeting dataset.

User ID
Creation time T
Post ID
Creation time of the retweeted or un-retweeted post
User ID of the retweeted or un-retweeted post
Post content
Retweeted or un-retweeted

**Table 2:** The confusion matrix for the binary classification problem.

	Label 0 (predicted)	Label 1 (predicted)
Label 0 (actual)	True positive	False negative
Label 1 (actual)	False positive	True negative

**Table 3:** The method comparisons of accuracy and compression rate.

	Accuracy	Compression ratio
KNN (*k* = 1)	0.754	0
KNN (*k* = 2)	0.863	0
CNN (*k* = 1)	0.712	0.418
CNN (*k* = 2)	0.732	0.397
ICKNN (*k* = 1)	0.734	0.634
ICKNN (*k* = 2)	0.836	0.427

**Table 4:** The method comparisons of time cost for classification.

Method	Time cost (s)	Percentage (decrease)
KNN	429	36%
CNN	420	28%
ICKNN	308	—

## Data Availability

The datasets can be obtained from the author upon request.
